# The Interplays between Autophagy and Apoptosis Induced by Enterovirus 71

This article has been retracted.

**DOI:** 10.1371/journal.pone.0056966

**Published:** 2013-02-20

**Authors:** Xueyan Xi, Xiaoyan Zhang, Bei Wang, Tao Wang, Ji Wang, He Huang, Jianwei Wang, Qi Jin, Zhendong Zhao

**Affiliations:** 1 MOH Key Laboratory of Systems Biology of Pathogens, Institute of Pathogen Biology, Chinese Academy of Medical Sciences and Peking Union Medical College, Beijing, China; 2 Department of Medical Laboratory Science, Fengyang College Shanxi Medical University, Shanxi, China; Karmanos Cancer Institute, United States of America

## Abstract

**Background:**

Enterovirus 71 (EV71) is the causative agent of human diseases with distinct severity, from mild hand, foot and mouth disease to severe neurological syndromes, such as encephalitis and meningitis. The lack of understanding of viral pathogenesis as well as lack of efficient vaccine and drugs against this virus impedes the control of EV71 infection. EV71 virus induces autophagy and apoptosis; however, the relationship between EV71-induced autophagy and apoptosis as well as the influence of autophagy and apoptosis on virus virulence remains unclear.

**Methodology/Principal Findings:**

In this study, it was observed that the Anhui strain of EV71 induced autophagy and apoptosis in human rhabdomyosarcoma (RD-A) cells. Additionally, by either applying chemical inhibitors or knocking down single essential autophagic or apoptotic genes, inhibition of EV71 induced autophagy inhibited the apoptosis both at the autophagosome formation stage and autophagy execution stage. However, inhibition of autophagy at the stage of autophagosome and lysosome fusion promoted apoptosis. In reverse, the inhibition of EV71-induced apoptosis contributed to the conversion of microtubule-associated protein 1 light chain 3-I (LC3-I) to LC3-II and degradation of sequestosome 1 (SQSTM1/P62). Furthermore, the inhibition of autophagy in the autophagsome formation stage or apoptosis decreased the release of EV71 viral particles.

**Conclusions/Significance:**

In conclusion, the results of this study not only revealed novel aspect of the interplay between autophagy and apoptosis in EV71 infection, but also provided a new insight to control EV71 infection.

## Introduction

Enterovirus 71 (EV71) was first identified and isolated from the feces of an infant suffering from encephalitis in 1969 in California [1]. Subsequently, EV71 was reported as the agent involved in severe neurological diseases such as meningitis, encephalitis, monoplegia and acute flaccid paralysis [2]. The virus was also associated with non-neurological diseases such as hand, foot and mouth disease (HFMD), herpangina and pulmonary edema [3]–[6]. Among young children, EV71 is a notable cause of central nervous system (CNS) disease that usually results in rapid clinical deterioration and death. However, due to the lack of understanding of its viral pathogenesis, there are no effective vaccines or antiviral therapies currently available for the control and prevention of its fatal outbreaks.

After the cells are infected with EV71, the cells go through the disease process until death. According to morphological changes during the process of cell death, the programmed cell death (PCD) was divided into three types including apoptosis, autophagy and programmed necrosis. Recently, more researches have been focused on the relationship of autophagy and apoptosis [7]–[11]. The functional relationship between autophagy and apoptosis is complex under certain circumstances. Autophagy constitutes a stress adaptation that avoids cell death, whereas in other cellular settings, it constitutes an alternative cell-death pathway [12]–[14]. Autophagy and apoptosis might be triggered by common upstream signals, which sometimes results in a combined autophagy and apoptosis. In other instances, the cell switches between the two responses in a mutually exclusive manner [15]. Apoptotic cell death is induced by inhibiting the accumulation of autophagosomes in various carcinoma cells [16], which suggests that the autophagic process prevents apoptotic cell death. However, some studies have demonstrated that the autophagy process can also induce apoptotic cell death [17]. As previously reported, EV71 virus induced the autophagy [18] as well as apoptosis [19]–[21]; however, the relationship between EV71 virus-induced autophagy and apoptosis remains unclear. Thus, unraveling this relationship could provide new clues to elucidate the pathogenesis of EV71 infection.

Reducing the viral particle release is an effective strategy to control virus infection. Wang et al. [22] demonstrated that when apoptosis was inhibited by Phyllaemblicin B, the viral virulence of coxsackie virus B3 was markedly inhibited. However, Ahn et al. [23] suggested that the caspase inhibitor significantly inhibited apoptosis with no influence on coxsackie virus production and cell death in Hela cells. In addition, Jackson et al. [24] demonstrated that the stimulation of autophagy increased poliovirus yield while its inhibition decreased it. Therefore, the influence of autophagy and apoptosis on EV71 viral particle release was studied by our group. Also, a process to decrease the EV71 viral particles by regulating the autophagy or apoptosis was evaluated, which could provide a new strategy for prevention and control of EV71 infection.

RD-A cells are a subset of cells that are often used for the proliferation and amplification of EV71. Anhui strain of EV71 is isolated from the throat swab of a child with severe HFMD, when HFMD broke out in Fuyang, Anhui Province, China in May 2008. The cells and the strain were selected in this study as a model to understand the impact of autophagy and apoptosis on viral replication. The autophagy and apoptosis induced by Anhui strain of EV71 in RD-A cells was examined. The relationship between the autophagy and apoptosis induced by EV71 was studied by either using chemical inhibitors or RNA interference against essential autophagic or apoptotic genes. Finally, the effect of autophagy and apoptosis on EV71 viral particle release was investigated.

## Results

### EV71 induced autophagy in RD-A cells

To determine if autophagy was induced by EV71 virus in RD-A cells, confocal microscopy was performed in EV71-infected cells (Fig. 1A). The RD-A cells were initially transfected with a green fluorescent protein (GFP) and microtubule-associated protein light chain 3 (LC3) fusion protein, a specific marker of autophagosomes, for 24 hours. These cells were then infected with EV71 virus (Anhui strain) at the Multiplicity of Infection (MOI) of 10. In contrast to the diffused expression pattern of GFP-LC3 in control cells, GFP-LC3 showed punctuated accumulation in the EV71 infected cells (Fig. 1A). The number of punctated GFP-LC3 in each cell was counted (at least 50 cells were included for each group). The EV71-infected cells showed an increased punctate staining of GFP-LC3 (Fig. 1A) (P<0.01).

**Figure 1:** EV71 induced autophagy in RD-A cells. (A) The LC3 punctate were detected by confocal microscopy. After transfected with GFP-LC3 plasmid for 24 h, the RD-A cells were infected with EV71 virus (Anhui strain) at MOI of 10. After 12 hours of infection, cells grown on coverslips were fixed with freshly prepared 4% paraformaldehyde for 15 minutes at room temperature. The anti-EV71 monoclonal antibody and TRITC-conjugant anti mouse IgG antibody were added. The coverslips with fixed cells were mounted into microscopy chamber and directly visualized in phosphate buffer. The fluorescence of GFP-LC3 was viewed, images were acquired through GFP channel and the dots of GFP-LC3 were counted. Data are shown as the mean of three independent experiments. The double asterisks denote significant difference (p<0.01). (B) The RD-A cells were infected by EV71 at different MOI for 12 hours. The cells were lyzed and Western blot were performed. (C) The RD-A cells were infected by EV71 at multiplicity of infection of 10, lyzed at different time points post infection, and then Western blot were performed. Results are representative of three independent experiments. (D) The RD-A cells were infected by EV71 at multiplicity of infection of 1, 5 and 10, lyzed at different time points (6 h, 9 h, 12 h and 24 h) post infection, and then Western blot were performed. Results are shown as histogram. The results are representative of two independent experiments.

The conversion of LC3-I to LC3-II is assumed to be an accurate indicator of autophagy [18]. Therefore, the expression of LC3 in RD-A cells that were exposed to EV71 virus was investigated. At the fixed infection time of 12 hours, EV71 induced the conversion of LC3-I to LC3-II in a dose dependent fashion (Fig. 1B). To detect the impact of infected EV71 on autophagic flux, the expression of sequestosome 1 (SQSTM1/p62), a selective substrate of autophagy, was measured. The level of P62 was decreased after the cells were infected with EV71, suggesting an enhanced autophagic flux (Fig. 1B). Meanwhile, at the fixed infection dosage (MOI = 10), EV71 virus increased the conversion of LC3-I to LC3-II as well as P62 degradation in a time-dependent manner (Fig. 1C). The change of LC3 and P62 at different infection dosages and infection time points was also detected. With an increase in the dosage and time course of infection, the conversion of LC3-I to LC3-II and the degradation of P62 increased accordingly (Fig. 1D). Based on these results, EV71 induced autophagy in RD-A cells.

### EV71 induced caspase-dependent apoptosis in RD-A cells

In this study, EV71-induced cell death was examined by ImageStream Multispectral Flow Cytometer. The data was analyzed using the ImageStream Data Analysis and Exploration Software (IDEAS). In the software, the apoptosis wizard provided the guide through the process of creating the features and graphs to measure apoptosis using the images of the nuclear dye and the bright field. The cells in R4 region presented in Fig. 2A were identified as apoptotic cells. The percentage of apoptotic cells was also shown in Fig. 2A. Visual confirmation of morphology was performed by clicking on the dots in the region in the appropriate locations. The EV71 induced apoptosis was further confirmed by Flow cytometry (Fig. 2B). The sum of the percentage in second quadrant and fourth quadrant was considered to be the percentage of apoptotic cells. These results demonstrated that EV71 infection caused an apparent apoptotic cell death in RD-A cells.

**Figure 2:** EV71 induced caspase-dependent apoptosis in RD-A cells. (A) RD-A cells infected with EV71 virus at the MOI of 0, 1, 5 and 10 for 12 h were trypsinized and harvested. The cells were washed with PBS and incubated with 7-AAD at 4°C for 30 minutes, detected by ImageStream multispectral flow cytometer and analyzed using the ImageStream Data Analysis and Exploration Software. Apoptotic cells are identified in R4 region. The percentage of apoptosis cells was listed in histogram. Visual confirmation of morphology was performed by clicking on dots in the region in the appropriate locations. (B) RD-A cells infected with EV71 virus at MOI of 0, 1, 5 and 10 were trypsinized and harvested. The cells were washed with PBS and incubated with a FITC-labeled Annexin V and stained with propidium iodide (PI) at room temperature for 15 minutes. The cells were analyzed on flow cytometer. The Annexin V-positive and PI-negative cells were considered to be apoptotic cells in early phase. The annexin V-positive and PI-positive cells were considered to be apoptotic cells in later phase. The percentage of apoptotic cells was also presented in histogram. Data are shown as the mean of three independent experiments. (C) The RD-A cells were infected by EV71 at different MOI for 12 hours. The cells were lyzed and Western blot were performed. (D) The RD-A cells were infected by EV71 at MOI of 10. The cells were lyzed at different time points post infection and Western blot were performed. Results are representative of three independent experiments.(E) The RD-A cells were infected by EV71 at multiplicity of infection of 1, 5 and 10, lyzed at different time points (6 h, 9 h, 12 h and 24 h) post infection, and then Western blot were performed. Results are shown as histogram. The results are representative of two independent experiments.

The ploy (ADP-Ribose) polymerase (PARP) and caspase-3 are believed as apoptosis hallmarks [25] and the cleavage of PARP and caspase-3 in RD-A cells that were exposed to EV71 virus was investigated. At a fixed infection time (12 hours), EV71 virus induced the cleavage of PARP and caspase-3 in a dose dependent manner (Fig. 2C). Meanwhile, at the fixed infection dosage (MOI = 10), EV71 virus induced the cleavage of PARP and caspase-3 in a time-dependent fashion (Fig. 2D). In addition, with the increase of the dosage and time course of EV71 infection, the cleavage of PARP and caspase-3 was increased accordingly (Fig. 2E). These results further demonstrated the occurrence of apoptosis in the RD-A cells that were infected with EV71.

At MOI of 10, both autophagy and apoptosis took place in the RD-A cells at 9 hours after infection with EV71. The most outstanding timing of both autophagy and apoptosis was 12 hours after infection. At 24 hours, cytopathic effect was remarkable and the cells were likely to undergo necrosis (data not shown). Therefore, in the rest of the studies, to explore the relationship between autophagy and apoptosis, the infection dose and infection time were set at 10 MOI and 12 hours, respectively.

### Inhibition of autophagosome formation decreased the apoptosis induced by EV71

To verify the relationship between the autophagy and apoptosis induced by EV71 in the early stages of autophagy, the cleavage of PARP and caspase-3 were detected after the infected cells were treated with chemical autophagy inhibitor or siRNA inference against autophagy related gene (Atg) 5 and Beclin1 gene. The cells were infected with or without EV71 and were co-cultured with different dosage of Wortmannin (an inhibitor of phosphoinositide 3-kinase (PI3K), which blocked autophagy at autophagosome formation stage). The cells were then collected and were applied to Western blot and flow cytometry analysis with fluorescein isothiocyanate (FITC)-Annexin V and Propidium iodide (PI). Upon EV71 infection, the inhibition of autophagy with Wortmannin decreased the cleavage of PARP and caspase-3 in a dose-dependent manner (Fig. 3A). Meanwhile, the inhibition of autophagy with Wortmannin decreased the number of apoptotic cells (Fig. 3B). In addition, using the RNA interference approach, it was found that the knockdown of Atg5 and Beclin1 remarkably reduced the cleavage of PARP and caspase-3 (Fig. 3C) along with decreasing the number of apoptotic cells (Fig. 3D).

**Figure 3.The:** inhibition of autophagosome formation decreased the apoptosis induced by EV71. (A) When RD-A cells infected with EV71 or without EV71 were co-cultured with different dosage of Wortmannin for 12 hours, the cells were lyzed and Western blot were performed. The results of western are representatives of the three independent experiments. The statistical analysis of PARP/Actin and caspase-3/Actin are the mean of three independent experiments. Mock value is set on 100% each experiment. (B) The RD-A cells treated as (A) were collected and stained with Annexin V-FITC and PI. The flow cytometry analysis was performed. The percentage of apoptotic cells were shown in the form of histogram. (C) RD-A cells were transfected with control, Atg5 and beclin1 siRNA for 36 hours, the cells were treated with EV71 at the MOI of 10 for 12 h before Western blot with the indicated antibodies. (D) RD-A cells treated as (C) were collected and stained with Annexin V-FITC and PI. The flow cytometry analysis was performed. The percentage of apoptotic cells were shown in the form of scatter plots.

Some previous reports [26], [27] suggested that UV radiation resistance-associated gene (UVRAG) formed two different complexes (UVRAG-Beclin1 and UVRAG-Bax), which regulated the balance between autophagy and apoptosis. So, the expression of UVRAG was detected in RD-A cells treated with Wortmannin upon EV71 infection. The results showed that the degradation of UVRAG induced by EV71 was dose- and time-dependent (Fig. 4A, 4B) and it could be inhibited by Wortmannin (Fig. 4C). In addition, one report [27] suggested that UVRAG interacted with Bax, which inhibited apoptotic stimuli-induced mitochondrial translocation of Bax, reduction of mitochondrial membrane potential, cytochrome release and activation of caspase-9 and -3. Our results demonstrated that with the degradation of UVRAG that could be inhibited by Wortmannin, the expression of Bax increased correspondingly (Fig. 4C).

**Figure 4:** The inhibition of autophagy at the autophagosome formation inhibited the apoptosis through the interaction of UVRAG and BAX. The RD-A cells were infected by EV71 at different MOI for 12 hours (A) and at multiplicity of infection of 10, lyzed at different time points post infection (B). The western blot for UVRAG was performed. (C) When RD-A cells infected with EV71 or without EV71 were co-cultured with different dosage of Wortmannin for 12 hours, the cells were lyzed and Western blot were performed. The UVRAG and BAX were detected using corresponding monoclonal antibody. Results are representative of three independent experiments.

### Inhibition of autophagosome and lysosome fusion promoted the EV71-induced apoptosis

Chloroquine (CQ) has been reported to inhibit lysosomal acidification and therefore prevent autophagy by blocking autophagosome fusion and degradation [28]. The CQ was used in this study to detect the effect of autophagy on EV71-induced apoptosis. The cells were infected with or without EV71 and were co-cultured with different dosage of CQ. The cells were then collected and submitted to Western blot and flow cytometry. It was found that the inhibition of autophagy with CQ promoted the cleavage of PARP and caspase-3 in a dose-dependent manner (Fig. 5A). Also, the inhibition of autophagy with CQ increased the number of apoptotic cells (Fig. 5B).

**Figure 5:** Inhibition of the fusion of autophagosome with lysosome promoted the apoptosis induced by EV71. (A) When RD-A cells infected with EV71 or without EV71 were co-cultured with different dosage of CQ for 12 hours, the cells were lyzed and Western blot were performed. The results of western are representatives of the three independent experiments. The statistical analysis of PARP/Actin and caspase-3/Actin are the mean of three independent experiments. Mock value is set on 100% each experiment. (B) RD-A cells treated as (A) were collected and stained with Annexin V-FITC and PI. The flow cytometry analysis was performed. The percentage of apoptotic cells were shown in the form of histogram. Data are shown as the mean of three independent experiments.

### Inhibition of the lysosomal protease inhibited the EV71-induced apoptosis

Pepstatin A and E64d, the inhibitors of lysosomal protease, were used to detect the effect of autophagy on apoptosis induced by EV71. The cells infected with or without EV71 and were co-cultured with different dosage of E64d and pepstatin A. The cells were then collected for Western blot and flow cytometry analysis. The inhibition of autophagy with E64d and pepstatin A decreased the cleavage of caspase-3 in a dose-dependent manner (Fig. 6A). Likewise, the inhibition of autophagy with E64d and pepstatin A decreased the number of apoptotic cells (Fig. 6B).

**Figure 6:** Inhibition of the lysosomal protease decreased the apoptosis induced by EV71. (A) When RD-A cells infected with EV71 or without EV71 were co-cultured with different dosage of E64d and pepstatin A for 12 hours, the cells were lyzed and Western blot were performed. The results of western are representatives of the three independent experiments. The statistical analysis of PARP/Actin and caspase-3/Actin are the mean of three independent experiments. Mock value is set on 100% each experiment. (B) RD-A cells treated as (A) were collected and stained with Annexin V-FITC and PI. The flow cytometry analysis was performed. The percentage of apoptotic cells were shown in the form of histogram. Data are shown as the mean of three independent experiments.

### Inhibition of apoptosis increased the conversion of LC3-I to LC3-II and degradation of P62

Z-VAD-FMK, a pan-caspase inhibitor, has been reported to block the caspase-dependent apoptosis [29]. In this study, the LC3 type conversion and P62 degradation were examined after inhibition of the EV71-induced apoptosis by Z-VAD-FMK. The results showed that inhibition of apoptosis by Z-VAD-FMK increased the conversion of LC3-I to LC3-II and the degradation of P62 in a dose-dependent fashion (Fig. 7A). Meanwhile, the inhibition of apoptosis by Z-DEVD-FMK, a caspase-3 inhibitor, also increased the conversion of LC3-I to LC3-II and the degradation of P62 in a dose dependent fashion (Fig. 7B). Using the RNA interference approach, it was found that knockdown of caspase-3 significantly increased the conversion of LC3 and P62 degradation (Fig. 7C). Zalckvar's report [10] suggested that the connection of Atg5 and caspase-3 played an important role in the autophagy and apoptosis. In order to clarify the impact of Atg5 to apoptosis, we detected the expression of Atg5 when casapase-3 was inhibited or knocked down. The results demonstrated that with the increase of Z-DEVD-FMK, the expression of Atg5 was also increased (Fig. 8A). When caspase-3 was knocked down, the expression of Atg5 also increased (Fig. 8B).

**Figure 7:** Inhibition of apoptosis increased the conversion of LC3-I to LC3-II and degradation of P62. When RD-A cells infected with EV71 or without EV71 were co-cultured with different dosage of Z-VAD-FMK (A) and Z-DEVD-FMK (B) for 12 hours, the cells were lyzed and Western blot were performed. (C) RD-A cells were transfected with control and caspase-3 siRNA for 36 hours, the cells were treated with EV71 at the MOI of 10 for 12 h before Western blot with the indicated antibodies. The results of western are representatives of the three independent experiments. The statistical analysis of LC3II/LC3I and P62/Actin are the mean of three independent experiments. Mock value is set on 100% each experiment.

**Figure 8:** Inhibition of apoptosis promoted the autophagy through the ATG5. (A) When RD-A cells infected with EV71 were co-cultured with different dosage of Z-DEVD-FMK for 12 hours, the cells were lyzed and Western blot were performed. (B) RD-A cells were transfected with control and caspase-3 siRNA for 36 hours, the cells were treated with EV71 at the MOI of 10 for 12 h for Western blot with ATG5 antibody. Results are representative of three independent experiments.

### Inhibition of autophagy in the autophagosome formation stage and apoptosis decreased EV71 viral particle release

To check the influence of autophagy and apoptosis on the viral particle release, cultural supernatants from EV71-infected RD-A cells under the action of different dosage of Wortmannin and Z-VAD-FMK were collected and subjected to virus titeration by using the TCID50 method. The results showed that with the increase of the dosage of Wortmannin (Fig. 9A) and Z-VAD-FMK (Fig. 9B), the viral particles released into the cultural supernatants decreased gradually. By taking advantage of RNA inference of Atg5 and caspase-3, it was also shown that the virus titer in the cultural supernatant was decreased as compared to that of the supernatant of the cells treated with control siRNA (Fig. 9C).

**Figure 9:** The inhibition of autophagy and apoptosis prevented EV71 viral particle from release. RD-A cells were infected with EV71 in the presence or absence of Wortmannin (A) and Z-VAD-FMK (B) for 24 hours. The culture supernatant was collected and TCID50 examination was performed. (C) RD-A cells were transfected with control and Atg5 and caspase-3 siRNA for 36 hours, the cells were treated with EV71 at the MOI of 10 for 12 h. The culture supernatant was collected and TCID50 examination was performed. Data are shown as the mean of two independent experiments.

### Cathepsins might participate in the interplay of autophagy and apoptosis in the fusion stage of autophagosome with lysosome and autophagy execution stage

Previous reports demonstrated that treatment with CQ led to a dramatic increase in cathepsin D [30], which promoted apoptosis through activating caspase pathway and modifying pro-apoptotic molecular BAX and BAK [31]. In order to check the role of cathepsin D in EV71 infected cells, the expression of cathepsin D was detected in RD-A cells that were infected with EV71 upon being treated with different dosage of CQ. The results showed that with the increase of CQ dosage, the expression of cathepsin D increased (Fig. 10A). In autophagy execution stage, pepstatin A, an inhibitor of cathepsins D [32], [33], and E64d, a cell permeable inhibitor of cathepsins B, H and L [34] were used to evaluate the effect of autophagy to apoptosis induced by EV71. We found that with the increase of E64d and pepstatin A dosage, the expression of cathepsin D and cathepsin B in RD-A cells infected by EV71 decreased (Fig. 10B). Based on these results and that from Fig. 5 and Fig. 6, it was suggested that the cathepsins might participate in the interplay of autophagy and apoptosis in the fusion stage of autophagosome with lysosome and autophagy execution stage.

**Figure 10:** The cathepsins might participate in the interplay of autophagy and apoptosis in the fusion of autophagosome with lysosome and autophagy execution stage. When RD-A cells infected with EV71 were co-cultured with different dosage of chloriquine (A) and E64d and pepstatin A (B) for 12 hours, the cells were lyzed and Western blot was performed. Results are representative of three independent experiments.

## Discussion

Many studies have shown multiple connections between the autophagic and apoptotic processes, and the two phenomena jointly sealing the fate of the cells. Autophagy is a catabolic pathway that is often characterized by the formation of double-membrane vesicles (autophagosomes) that engulf cytoplasmic organelles and proteins and fuse with lysosomes in the end, which degrade their luminal content. Autophagy acts as a cytoprotective mechanism, favoring stress adaptation to avoid cell death [35], [36]. Apoptosis is programmed cell death and leads to the rapid demolition of cellular structures and organelles. When this process culminates in cellular shrinkage with nuclear chromatin condensation and nuclear fragmentation, it complies with the morphological definition of apoptosis [37]. Shimizuet al. [38] demonstrated that autophagy related to apoptosis by acting as a partner, an antagonist or an enabler of apoptosis depending on the cell type, stimulus and environment. In this study, in order to clarify the interplay of autophagy and apoptosis in EV71 infection in RD-A cells, apoptosis and autophagy were detected when the autophagy and apoptosis were inhibited by either a chemical inhibitor at different stages or by a single knockdown of essential genes through RNA interference; respectively. We ruled out the role of various single inhibitors on RD-A cells and provided the interaction possibility between autophagy and apoptosis under the action of various inhibitors in EV71 infection. During the course of EV71 infection in RD-A cells, the crosstalk between autophagy and apoptosis was very complex. In this study, it was demonstrated that the inhibition of EV71 induced autophagy at autophagosome formation and autophagy execution stages that might inhibit apoptosis. However, inhibition of autophagy at the stage of autophagosome and lysosome fusion might promote the apoptosis and the inhibition of EV71-induced apoptosis contributed to the autophagy. We summarized these findings in a brief chart about the relationship of autophagy and apoptosis in Fig. 11. In addition, the inhibition of autophagy or apoptosis by either chemical inhibitors or RNA interference decreased the release of EV71 viral particles.

**Figure 11:** The brief chart about the interplays of autophagy and apoptosis.

EV71 is a single, positive-stranded RNA virus that belongs to the Picornaviridae family [39]. The 7.4-kb genome of EV71 encodes a single polyprotein that is proteolytically cleaved to various structural and nonstructural viral proteins. In order to illustrate the contribution of the different viral components to both host autophagy and apoptosis pathway, we transfected the structural proteins of VP1, VP2, VP3 and VP4 and non-structural proteins or protein intermediate of 2A, 2B, 2C, 3A, 3AB, 3C and 3D into 293T cells. The cells were then subjected to autophagy and apoptosis detection by checking the LC3 conversion, p62 degradation and PARP cleavage. Due to the low transfection efficiency in RD-A cells (data not shown), these experiments were carried out in 293T cells. The results were shown in Fig. S1. It was found that none of the structural and non-structural proteins of EV71 separately induced a significant autophagy and apoptosis like the viral particles. This observation suggested that the induction of both autophagy and apoptosis might depend on a comprehensive interaction among the structural and non-structural proteins of EV71 in its life cycle in the host cells.

In the study, we also explored the possible mechanism of the interplay between autophagy and apoptosis according to the current results. The preliminary mechanism was presented in Fig. 11.

Wortmannin has been proposed to suppress the autophagosome formation by inhibiting the class III PI3K to block the production of PI3P, which is essential for the initiation of autophagy via recruitment of other ATG proteins at the isolation membrane or phagophore [40]. To explore the mechanism that the inhibition of autophagy by Wortmannin inhibited apoptosis, we detected the UVRAG, which regulated the balance between autophagy and apoptosis by two different complexes (UVRAG-Beclin1 and UVRAG-Bax) [26]. UVRAG interacted with Bax [27], which inhibited apoptotic stimuli-induced mitochondrial translocation of Bax, reduction of mitochondrial membrane potential, cytochrome release and activation of caspase-9 and -3. The results in our study also showed that the degradation of UVRAG was inhibited by Wortmannin, and the expression of Bax increased correspondingly (Fig. 4C). It provided a potential mechanism for the Wortmannin-inhibited autophagy that leads to an increased UVRAG and Bax expression in order to inhibit the apoptosis (Fig. 11). Definitely, an in-depth study is needed next to address the specific mechanisms of UVRAG and Bax in the interaction between autophagy and apoptosis.

Our results also showed that when the EV71-induced apoptosis was inhibited by Z-VAD-FMK (pan-caspase inhibitor), the RD-A cells treads to autophagy (Fig. 7A). This was consistent with the previous report of Sirois [41] highlighting that ZVAD-FMK negatively impacted autophagic vacuole (AV) maturation, possibly through preventing the release of AV components in the extracellular milieu and increasing the mean distance between AV and the cell membrane. Meanwhile, these results were corroborated caspase-3 inhibitor (Z-DEVD-FMK) caspase-3-deficient mice. It was observed that caspase-3 was an important regulator in autophagosome maturation. This encouraged us to detect the role of caspase-3 in the relationship of autophagy and apoptosis. As shown in Fig. 7B and 7C, the RD-A cells tend to undergo autophagy when they were treated with caspase-3 inhibitor (Z-DEVD-FMK) or caspase-3 was knocked down. In addition, by applying computational tools that are based on mining the protein–protein interaction database, a novel biochemical pathway between Atg5 and caspase-3 was obtained [10]. In order to clarify the impact of Atg5 on apoptosis in this study, the expression of Atg5 was detected when caspase-3 was inhibited or knocked down. The results demonstrated that with an increase in Z-DEVD-FMK, there was an increased expression of Atg5 (Fig. 8). Taken together, the co-relation of autophagy (in the autophagosome formation stage) and apoptosis was assumed to be related to ATG5 and caspase-3. When ATG5 was inhibited, the caspase-3 was also inhibited, thus inhibiting the apoptosis. Likewise, when caspase-3 was inhibited, ATG5 was activated, thus promoting the autophagy (Fig. 11). We are conducting an in-depth study of the role of the interaction between ATG5 and caspase-3 on the autophagy and apoptosis.

It was found that the inhibition of autophagosomes and lysosome fusion of by CQ promoted the apoptosis (Fig. 5). CQ is a weak alkali that can inhibit lysosomal acidification, which prevents the fusion of autophagosomes with lysosomes and subsequently leads to autophagic degradation. Carew et al. demonstrated that the treatment with CQ led to a dramatic increase in cathepsin D [30], which was active at physiologcal pH and promoted apoptosis through two aspect of action including activating caspase pathway and modifying pro-apoptotic molecular BAX and BAK [31]. Our results were consistent with the above report, where CQ inhibited EV71-induced autophagy and promoted the apoptosis of RD-A cells by activating cathepsin D (Fig. 10A). Another possibility was that the inhibition of autophagy might have resulted in a bioenergetic shortage which triggered apoptosis [42]. In a more subtle fashion, inhibition of autophagosome and lysosome fusion might subvert the capacity of cells to remove damaged organelles or misfolded proteins, which in turn would favor apoptosis.

In autophagy execution stage, pepstatin A (an inhibitor of cathepsins D) [32], [33] and E64d (a cell permeable inhibitor of cathepsins B, H and L) [34] were used to evaluate the effect of autophagy to apoptosis induced by EV71. Motyl et al. [43] suggested that inhibition of cathepsins by E64d significantly reduced the apoptotic cell number. Cathepsins, particularly cathepsin B, could be involved in the molecular switch between autophagy and apoptosis. Furthermore, it was found that E64d and pepstatin A inhibited EV71-induced autophagy and decreased the RD-A cells apoptosis by inhibiting cathepsin D and B (Fig. 10B). In the late stage of autophagy (the fusion of autophagosome with lysosome and autophagy execution stage), the role of CQ, E64d and pepstatin A seems to be linked through cathepsins.

Taken together, the inhibition of autophagy by Wortmannin inhibited the EV71-induced apoptosis possibly through increasing the expression of UVRAG thus impact on UVRAG and BAK interaction. The inhibition of apoptosis by Z-DEVD-FMK promoted the EV71-induced autophagy possibly through activating ATG5. In the fusion stage of autophagosome with lysosome, the inhibition of autophagy promoted the apoptosis in RD-A cells by activating cathepsins D. And the inhibition of autophagy in the execution stage inhibited the apoptosis by inhibiting cathepsin D and cathepsin B.

In this study, we also explored the role of the interplay between autophagy and apoptosis in viral particle release. It seems that influence of autophagy at different stages of autophagy development on EV71 viral particles release was achieved through the effect on the apoptosis The autophagy at the stage of autophagosome formation was inhibited by Wortmannin, the viral particle released was also inhibited (Fig. 9). Although autophagy during the stage of autophagosome formation might not have a direct impact on the virus release, it probably had an inhibitory effect on virus release through apoptosis inhibition. We did not check into the viral particles release at the fusion stage of autophagosome with lysosome and execution stage. But we might speculate that EV71 might have prompted the release of viral particles through concomitantly induced apoptosis at the fusion stage. And during the execution stage, viral particles release might reduce due to the inhibition of apoptosis. In addition, the apoptosis was inhibited by Z-VAD-FMK, the viral particle released was also inhibited (Fig. 9). Therefore, the information should be potentially helpful for the selection of inhibitors used to control EV71 viral particle release as a potential strategy for prevention and control of EV71 infection.

## Materials and Methods

### Cell culture and virus propagation

Human rhabdomyosarcoma (RD-A; ATCC, CCL-136) cells were maintained in L-glutamine containing Dulbecco's modified Eagle's medium (DMEM) (Hyclone) supplemented with 10% fetal bovine serum (FBS) (Gibco) plus penicillin/streptomycin (200 U/ml), and cultured at 37°C in a 5% CO_2_ incubator. At 80% confluence, cells were trypsinized with 0.25% trypsin (Solarbio) and sub-cultured in the complete medium. Virus infection was carried out as follows. Briefly, RD-A cells were infected with EV71 at the indicated multiplicity of infection (MOI). Viruses were washed away after 2 hours, cells were then cultured with fresh medium supplemented with 2% FBS. At the indicated time points post infection, the cells and culture supernatant were harvested.

### Chemicals and antibodies

The antibodies to Pepstatin A (Sigma-Aldrich, P5318), E64d (Sigma-Aldrich, E8640), β–actin (Sigma-Aldrich, A5316), ATG 5 (Sigma-Aldrich, A0731) and polyclonal antibodies of LC3 (Sigma-Aldrich, L7543) were purchased from Sigma-Aldrich; Z-VAD-FMK (R&D, FMK001) was purchased from R&D systems; antibodies against UVRAG (CST, 5320), caspase-3 (CST, 9662) and PARP (CST, 9542) were obtained from Cell Signaling; antibodies to P62 (Santa Cruz, sc-28359) and beclin 1 (Santa Cruz, sc-11427) were purchased from Santa Cruz Biotechnology; anti-EV71 (Millipore, MAB979) antibody was got from Millipore; Chloroquine and Z-DEVD-FMK were purchased form MBL Company.

### Plasmids and siRNAs

GFP-LC3 plasmid was a kind gift of Dr. Xuejun Jiang (Biological Resource Center of Institute of Microbiology; Chinese Academy of Sciences). To construct plasmids VP1, VP2, VP3, VP4, 2A, 2B, 2C, 3A, 3AB, 3C, and 3CD, fragments of EV71 cDNA were cloned into the HindIII and SalI sites of pEGFPC1 vector, resulting in GFP fusion proteins. The siRNA specific for Caspase-3 (Santa Cruz, sc-29437), Atg5 (Santa Cruz, sc-41445) were purchased from Santa Cruz Biotechnology along with the control siRNA. siGENOME SMART pool of BECN1 (8678) targeting Beclin 1 was bought from Dharmacon.

### Confocal microscopy

RD-A cells were transfected with GFP-LC3 expressing plasmid, after 24 hours of transfection, cells were infected with EV71 virus at indicated MOI. After 12 hours, cells grown on coverslips were fixed with freshly prepared 4% paraformaldehyde for 15 minutes at room temperature. The anti-EV71 antibody (Millipore, MAB979) and TRITC-conjugant anti mouse IgG antibody (Zhongshan, ZF-0313) was incubated. The coverslips with fixed cells were mounted into confocal microscopy (Leica, TCSSP5) and directly visualized in phosphate buffer. The fluorescence of GFP-LC3 was viewed, imaged and the dots of GFP-LC3 were counted.

### Western blot

Cells were lyzed in buffer containing 150 mMNaCl, 25 mMTris (pH 7.4), 1% NP-40, 0.25% sodium deoxycholate, and 1 mM EDTA as well as a proteinase inhibitor cocktail (Roche). Lysed cells were electrophoresed on 12% SDS-PAGE and transferred to polyvinylidene fluoride membranes (BioRad). The membranes were blocked with 5% dried skimmed milk and then incubated with corresponding antibodies at 4°C overnight. This was followed by incubation with the corresponding IRDye Fluor 800-labeled IgG or IRDye Fluor 680-labeled IgG secondary antibody (Li-Cor Bioscience). After the membranes were washed with 0.1% Tween20 in PBS, the signal were scanned by using an Odyssey Infrared Imaging System (Li-Cor Bioscience) at a wavelength of 700 nm to 800 nm and analyzed with Odyssey software. The molecular sizes of the developed proteins were determined by comparison with pre-stained protein markers (New England Biolabs). Several western bands were analyzed to verify the linear range of the chemiluminescence signals and the quantifications were carried out using Quantity One software.

### ImageStream multispectral flow cytometer

RD-A cells infected with EV71 virus at the MOI of 0, 1, 5 and 10 for 12 h were trypsinized and harvested. The cells were washed with PBS and incubated with 7-AAD (Invitrogen) at 4°C for 30 minutes and then analyzed on ImageStream multispectral flow cytometer (Amnis). An ImageStream multispectral imaging flow cytometer works similar to classical flow cytometer except that it also allows visualization of individual cells passing through its flow chamber. The snapshots of each cell provided additional information of cellular morphology and spatial distribution. The data was analyzed using the ImageStream Data Analysis and Exploration Software (IDEAS).

### Flow cytometry

For flow cytometry analysis, RD-A cells that were infected with EV71 or without EV71 co-cultured with autophagy and apoptosis inhibitor. The cells were collected, washed with PBS and incubated with a FITC-labeled annexin V and stained with PI (Baosai Biotech) at room temperature for 15 minutes and then analyzed on flow cytometer (BD CantoII). The annexin V-positive/PI-negative cells were considered to be apoptotic cells at the early period, annexin V-positive/PI-positive cells were considered to be apoptotic cells at the later period, whereas PI-single positive cells were considered necrotic.

### TCID50 (50% tissue culture infective dose)

The titer of virus was calculated with TCID50. The virus particle in cell culture supernatant were collected by centrifugation at 4000 rpm for 5 minutes at 4°C. 5000 cells/well were put in 96 wells plate in DMEM medium plus 2% FBS before 1 day. The determined virus suspension were diluted with DMEM medium plus 2% FBS by 10-fold of serial dilutions from 10^−1^ to 10^−8^. 100 µl of each dilution was transfered to the plate with cells to make total of 200 µl per wells. The cells were cultured at 37°C for 5 days and cells were observed daily. The TCID50 was calculated according to the Behrens-Kärber formula: log TCID50 = L-d (S −0.5), where: L = lowest log dilution values used in the experiment; d = log value of the dilution gradient; S = the sum of the positive parts.

### Statistics analysis

The statistical comparisons were performed by using Student's t test. Value of P<0.05 was considered statistically significant.

## Supporting Information

Figure S1 **None of the structural and non-structural proteins of EV71 separately induced a significant autophagy and apoptosis.** The plasmid pEGFPC1 containing VP1,VP2, VP3, VP4, 2A, 2B, 2C, 3A, 3AB, 3C, and 3CD were transfected into 293T cells for 36 h, the cells were lyzed and Western blot for LC3, P62, PARP, GFP and β-actin was performed.
(TIF)
